# Stacking Ensemble Method for Gestational Diabetes Mellitus Prediction in Chinese Pregnant Women: A Prospective Cohort Study

**DOI:** 10.1155/2022/8948082

**Published:** 2022-09-13

**Authors:** Ruiyi Liu, Yongle Zhan, Xuan Liu, Yifang Zhang, Luting Gui, Yimin Qu, Hairong Nan, Yu Jiang

**Affiliations:** ^1^Department of Epidemiology and Biostatistics, School of Population Medicine and Public Health, Chinese Academy of Medical Sciences and Peking Union Medical College, Beijing, China; ^2^School of Public Health, LKS Faculty of Medicine, The University of Hong Kong, Hong Kong, China; ^3^Department of Endocrinology, Shenzhen Longhua Maternity and Child Healthcare Hospital, Shenzhen, China

## Abstract

Gestational diabetes mellitus (GDM) is closely related to adverse pregnancy outcomes and other diseases. Early intervention in pregnant women who are at high risk of developing GDM could help prevent adverse health consequences. The study aims to develop a simple model using the stacking ensemble method to predict GDM for women in the first trimester based on easily available factors. We used the data from the Chinese Pregnant Women Cohort Study from July 2017 to November 2018. A total of 6,848 pregnant women in the first trimester were included in the analysis. Logistic regression (LR), random forest (RF), and extreme gradient boosting (XGBoost) were considered as base learners. Optimal feature subsets for each learner were chosen by using recursive feature elimination cross-validation. Then, we built a pipeline to process imbalance data, tune hyperparameters, and evaluate model performance. The learners with the best hyperparameters were employed in the first layer of the proposed stacking method. Their predictions were obtained using optimal feature subsets and served as meta-learner's inputs. Another LR was used as a meta-learner to obtain the final prediction results. Accuracy, specificity, error rate, and other metrics were calculated to evaluate the performance of the models. A paired samples *t*-test was performed to compare the model performance. In total, 967 (14.12%) women developed GDM. For base learners, the RF model had the highest accuracy (0.638 (95% confidence interval (CI) 0.628–0.648)) and specificity (0.683 (0.669–0.698)) and lowest error rate (0.362 (0.352–0.372)). The stacking method effectively improved the accuracy (0.666 (95% CI 0.663–0.670)) and specificity (0.725 (0.721–0.729)) and decreased the error rate (0.333 (0.330–0.337)). The differences in the performance between the stacking method and RF were statistically significant. Our proposed stacking method based on easily available factors has better performance than other learners such as RF.

## 1. Introduction

Gestational diabetes mellitus (GDM) is defined as glucose intolerance with onset or first recognition during pregnancy [1]. Worldwide, the prevalence of GDM varies geographically and ethnically, ranging from 1% to more than 30%. Middle Eastern countries and some North African countries have the highest GDM prevalence, followed by Southeast Asia and the Western Pacific region. In the Western Pacific region, the prevalence of GDM in Chinese women is significantly higher than in other countries [2]. Meanwhile, Asian women are at higher risk than other ethnic groups [3, 4]. GDM is significantly associated with short-term and long-term health consequences for mother and offspring [2]. High maternal glucose levels may increase the risk of pregnancy complications and adverse pregnancy outcomes such as preeclampsia, polyhydramnios, and macrosomia. According to earlier studies, women with GDM were more likely to develop metabolic syndrome (e.g., type 2 diabetes, adiposity, hypertension, and dyslipidaemia), cardiovascular disease (e.g., ischaemic heart disease and stroke), kidney disease, and retinal disease [5–9]. In particular, women with a history of GDM have a nearly 10-fold higher risk of type 2 diabetes than women with normoglycemic pregnancy [10]. For offspring, GDM is also associated with an increased risk of childhood obesity [11] and glucose intolerance [12].

Generally, GDM screening is recommended at 24–28 weeks of gestation. However, evidence has shown that a high glucose concentration in early pregnancy may increase the risk of adverse pregnancy outcomes [13]. Therefore, early screening for GDM can be beneficial because identifying women who are at high risk of GDM during the first trimester may have sufficient time to allow early intervention and reduce the occurrence of GDM or other related diseases. Several predictive models have been developed in earlier research studies to aid in the screening of women who are at risk of developing GDM. Single learners like logistic regression (LR), k-nearest neighbor (KNN), support vector machine (SVM), and deep neural network (DNN), as well as ensemble learning techniques like random forest (RF) and extreme gradient boosting (XGBoost), are frequently used algorithms in GDM prediction [14–16]. Recently, researchers started to focus more on the performance of ensemble learning in the prediction of GDM as compared to a single learner. Bagging and boosting are two popular ensemble learning techniques, but they are often used to integrate homogeneous base learners, such as decision tree (DT). Stacking is a suitable method for integrating different types of base learners, which is less used in GDM prediction. Kumar et al. proposed a stacked ensemble model with a gradient boosting classifier and SVM for predicting GDM risk, and their method achieved great performance with an AUC of 0.93 [17]. Their results demonstrated the effectiveness of stacking methods, but they used biochemical factors such as HbA1c, fasting insulin, and triglycerides/HDL ratio. Although various clinical indicators are important for predicting GDM, they are often difficult to obtain in areas with poor healthcare resources. Only a few studies have explored prediction models based solely on self-reported sociodemographic and behavior-related data. Nevertheless, constructing pregnancy-related predictive models based on these data is more feasible and practical in areas of severe shortage [18]. It is necessary to further explore the feasibility of constructing GDM prediction models based on easily available predictors such as age, weight, lifestyle, and disease history.

We aim to build a simple model for predicting the risk of GDM in women in the first trimester based on stacking methods and easily available predictors. We also use data from a prospective cohort study of pregnant women to collect health-related information on sociodemographic characteristics, physical measurements, lifestyle, behavioral factors, environmental factors, and more. The importance of these factors in different machine learning models is explored to provide some basis for future research.

### 1.1. Related Works

In the past few decades, machine learning algorithms have been used in various healthcare domains. Shamshirband et al. [19] discussed the applications of state-of-the-art machine learning approaches in healthcare systems. Some mainstream machine learning algorithms, especially the DNN, convolutional neural network (CNN), recurrent neural network (RNN), deep belief network (DBN), autocoding (AE), and other deep learning algorithms, have been applied to speech recognition, drug discovery, disease detection, computer vision, target detection, natural language processing, and other fields. In addition, some researchers have refined machine learning techniques for the prediction and identification of genetic sites and sequences, the prediction of COVID-19 pandemic outcomes, disease detection based on images, the construction of smart healthcare systems, and clinical expert systems. Chen et al. [20] and Zou et al. [21] reported different ensemble methods based on the CNN and long short-term memory (LSTM) to predict the human N6-methyladenosine sites from mRNA sequences. Deif et al. [22] came up with a deep bidirectional recurrent neural networks (BRNNs) model that combined with LSTM and GRU to distinguish between the genome sequence of SARS-CoV-2 and other coronavirus strains. Kumar et al. [23] constructed two models for predicting COVID-19 by using modified LSTM and reinforcement learning algorithms. Qummar et al. [24] reported a deep learning ensemble approach for diabetic retinopathy detection based on fundus images. Lv et al. [25] presented a new interactive smart healthcare prediction and evaluation model based on deep learning algorithms. Sadeghipour et al. [26] proposed an expert clinical system by using the XCSR classifier for diagnosing obstructive sleep apnea. This group of researchers also developed an intelligent system for diagnosing diabetes based on the XCSLA system [27].

Diabetes is one of the most common chronic noncommunicable diseases and consists of three main types: type 1 diabetes, type 2 diabetes, and GDM. Diabetes is strongly associated with lifestyle behaviors, unhealthy diets, and other factors, and early intervention in these modifiable risk factors is of great importance. Early intervention can prevent more serious disease outcomes in people with diabetes or reduce the risk of developing diabetes in those who are at risk. Machine learning techniques have been demonstrated to be effective in the early diagnosis and prevention of diabetes [28]. Traditional machine learning techniques such as LR, DT, SVM, NB, and KNN have been used for the classification and prediction of diabetes in the past few years [29]. Kumar et al. [30] proposed a multifaceted approach based on electronic health records of diabetic patients to simultaneously identify type 1 diabetes, type 2 diabetes, and GDM. They were using RF, LDA, SVM, KNN, and CART algorithms to learn the data patterns and predict diabetes. The result showed that RF was the most suitable algorithm for this dataset and had high accuracy in the classification of different types of diabetes. For binary classification, Ye et al. [31] used data from a single-centre and retrospective cohort study to compare the performance of various statistical methods and machine learning algorithms in GDM prediction. They used eight machine learning algorithms, including Gradient Boosting Decision Tree (GBDT), AdaBoost, LGB, LR, Vote, XGBoost, DT, RF, and two common regressions, including stepwise LR and LR with RCS. In this study, researchers performed data preprocessing steps such as missing value imputation and data standardization. The features of the included models were screened according to the Pearson correlation coefficient, and undersampling was performed to deal with imbalanced data. GBDT was considered to be the most effective machine learning algorithm, with an average AUC of 0.74.

In general, ensemble methods had better performance than single learner. Ensemble learning is a promising field, mainly including bagging, boosting, and stacking. Bagging and boosting methods are widely used, such as RF, GBDT, AdaBoost, XGBoost, and so on. These two kinds of methods mainly integrate the same type of weak learner to form a new strong learner. Whereas, stacking methods are applied to different base learners and emphasize the heterogeneity between base learners. The heterogeneity among base learners includes not only the use of different machine learning algorithms but also the application of different feature subsets and hyperparameter combinations [32, 33]. Ekbal et al. [34] developed a stacking method for entity extraction based on a different subset of features. They used genetic algorithms to select the optimal feature subset of SVM and conditional random field (CRF) models, respectively, and developed SVM and CRF models based on their feature subsets. The trained SVM and CRF models were used as base learners for stacking methods. Their methods had higher performance in the GENETAG and GENIA benchmark datasets, with F-measure values of 94.70% and 75.17%, respectively. However, more evidence is needed on the effectiveness of this approach in the prediction and classification of diabetes, especially GDM.

What is more, how to reduce dimension and select the optimal feature subset is an important step. Filter methods, wrapper methods, and embedded methods are three main feature selection techniques. Filter methods are based on feature correlation, such as Pearson correlation coefficient, ANOVA, chi-square, and so on. Both the wrapper method and the embedded method depend on the algorithm, and the feature subset that is most suitable for the model is selected by the coefficient or feature importance. At present, some researchers believe that the use of a single feature selection method has certain limitations. Therefore, He et al. [35] proposed a feature ranking and dimensionality reduction tool, MRMD 2.0, which takes into account multiple feature selection methods and is suitable for datasets in different situations.

## 2. Materials and Methods

### 2.1. Data Source and Participants

The data used in the present study were obtained from the Chinese Pregnant Women Cohort Study (CPWCS), which is a multicentre prospective cohort study. A total of 24 hospitals from 15 representative provinces in China were involved in the CPWCS, including Beijing, Shandong, Sichuan, Chongqing, Xinjiang, Jilin, Henan, Shanxi, Jiangxi, Jiangsu, Guizhou, Inner Mongolia, Guangdong, Anhui, and Hunan. From July 25, 2017, to November 26, 2018, 9,193 pregnant women at 5–13 weeks of gestation were recruited. Of them, 2,345 pregnant women without GDM data were excluded, leaving 6,848 eligible participants for final analyses (Figure 1). Additional information about the CPWCS has been reported in previous studies [36, 37].

### 2.2. Ethics Statement

All of the participants were provided with written informed consent for inclusion before they participated in the study. The study was approved by the Ethics Review Committee at the Department of Scientific Research, Peking Union Medical College Hospital (approval number: HS1345). The study is registered at ClinicalTrials.gov (NCT03403543).

### 2.3. Definition of GDM

In accordance with the International Association of Diabetes and Pregnancy Study Group criteria, a 75 g oral glucose tolerance test at 24–28 gestational weeks was employed for GDM screening. GDM was diagnosed if any of the following conditions were met: a fasting plasma glucose (PG) concentration of ≥5.1 mmol/L, a 1-hour PG concentration of ≥10.0 mmol/L, or a 2-hour PG concentration of ≥8.5 mmol/L.

### 2.4. Features of the Prediction Model

Easily available factors such as sociodemographic, behavioral, and environmental factors were used to construct the model. Baseline information on pregnant women was collected through self-administered questionnaires, including personal information, such as maternal age, body mass index (BMI) before pregnancy, personal and household annual income, education level, and environmental exposures; behavioral factors, such as physical activity, tobacco consumption, and alcohol consumption; dietary habits, including intake of unsaturated fatty acids and dietary supplements; depression level; sleep quality; family history; abortion history; gynecological disease history; and internal disease history.

Maternal age was categorized into three groups: <25, 25–30, and >30 years. BMI before pregnancy was categorized into three groups: <18.5, 18.5–24.0, and >24.0 kg/m^2^. Levels of education included primary school and below, junior and senior high school, university, and master's degree and above. Personal annual income was divided into three levels using the boundaries of 50,000 CNY and 100,000 CNY, and household annual income was divided into three levels using the boundaries of 100,000 CNY and 200,000 CNY. The level of physical activity of pregnant women was classified by its intensity (vigorous, moderate, or mild).

The participants' dietary habits were assessed using the qualitative food frequency questionnaire (Q-FFQ) [38]. The Q-FFQ covered 17 major food groups: roughage, tubers, vegetables, fruit, meat, poultry, seafood, fish, eggs, dairy products, soybean milk, other soybean products, nuts, fried food, western fast food, dessert, and puffed food [36]. In this study, each food group had eight frequency levels of habitual consumption (never, 1, 2, 3, 4, 5, or 6 days per week, or daily) during the previous week. The eight consumption levels were assigned a score of 1–8. Fried foods, Western fast foods, desserts, and puffed foods were among the food groups that scored 8–1, with a higher score representing a lower frequency of intake. The rest of the food groups scored 1–8, with a higher score representing a higher frequency of intake. The scores for all of the food groups were summed up to obtain the dietary habit score of each participant. The dietary habits were classified into four categories based on quartiles: poor (Q-FFQ score of ≤49), general (Q-FFQ score of 50–57), better (Q-FFQ score of 58–66), and best (Q-FFQ score of ≥67).

The depression level was measured using the Edinburgh Postnatal Depression Scale (EPDS) [39]. The depression level score was calculated for each participant according to the scoring rules of the scale, and an EPDS score of ≥13 was considered to indicate possible depression during pregnancy.

Information on the participants' sleep quality was collected using the Pittsburgh Sleep Quality Index (PSQI) [40]. The PSQI consists of seven components: subjective sleep quality, sleep latency, sleep duration, habitual sleep efficiency, sleep disturbances, use of sleeping medication, and daytime dysfunction, with a total of 19 individual items. The sum of the scores for the seven components was calculated for each participant, with a higher score indicating worse sleep quality. Sleep quality was classified according to the score achieved: poor (PSQI score of 16–21), general (PSQI score of 11–15), better (PSQI score of 6–10), and best (PSQI score of 0–5).

### 2.5. Data Preprocessing

Outliers can have a major impact on the performance of machine learning models. First, we dealt with the outliers in all independent features. Outliers were identified using the quartile range (IQR) approach. The difference between the third quartile (*Q*3) and the first quartile (*Q*1) is the IQR. Outliers were defined as values greater than *Q*3 + (1.5 ^*∗*^ IQR) or less than *Q*1 − (1.5 ^*∗*^ IQR) in this study. Then, using exploratory data analysis, we identified several inaccurate values as outliers. All outliers in different features were replaced with missing values and will be deemed missing values for filling, according to the above definition of outliers.

Eleven features with more than 15% of missing values were excluded from the models. The features with fewer missing values (≤15%) were filled using multiple imputation (MI). MI is an accurate method of filling in missing values and is recommended for use in studies to construct predictive models [41, 42]. After missing data processing, all of the continuous features, including age, BMI, personal annual income, and household annual income, were discretized into two or more categories. The diet score, depression score, and sleep quality score were calculated using the Q-FFQ, EPDS, and PSQI, respectively, and three categorical features were constructed. A total of 106 categories were included in the subsequent model building as predictors.

### 2.6. Feature Selection

The fundamental goal of feature selection is to find the optimal feature subset to optimize the machine learning algorithms' performance. In this study, we implemented recursive feature elimination cross-validation (RFECV) methods [43, 44] based on LR, RF, and XGBoost algorithms. RFE is the representative method of the wrapped method. This approach relies on specific attributes of the algorithm (such as coefficients and feature importance). In the present study, we applied 3-fold cross-validation to obtain the feature importance ranking of each model. For each feature, its importance score in each fold dataset was calculated, and the mean value was computed. The subset of features with the highest AUC value and the lowest number of features was considered to be the best. To ensure that the best combination of features was applicable to the model, LR, RF, and XGBoost algorithms were combined with RFECV, respectively. The features selected by each algorithm were used in the subsequent construction of a model based on that algorithm.

### 2.7. Base Learners' Development

For the LR model, we processed the features through a sigmoid function and output a prediction probability, which was transformed into a binary output, and the parameters of each feature were calculated using the maximum likelihood method [31]. In this study, the regularization mode (penalty) and degree (C) of the LR algorithm will be adjusted to optimize its performance.

The RF approach is an ensemble learning algorithm based on bagging. The principle is to use different random samples to train multiple decision trees and use the voting method to obtain the final classification result. Compared with the single decision tree, random forest is more robust, less likely to overfit, and usually has better performance. Bagging is mainly used for the integration of weak classifiers with great heterogeneity, which is a parallel ensemble method. In a given dataset containing *m* samples, random sampling is carried out in the way of putting them back. After *m* times of random sampling, *T* training sets containing *m* samples are obtained. Multiple base learners are trained based on these training sets, and then, the results of these base learners are combined. In the present study, the three parameters, including the number of trees in the forest (n_estimators), the maximum depth of the tree (max_depth), and the minimum number of samples required to split an internal node (min_samples_split), were searched in a specific searching space, and the best combination within this space was obtained to optimize the RF model.

XGBoost is an efficient and extensible ensemble learning classifier that is based on boosting, which is a further improvement to the GBDT, and the base learner of the XGBoost algorithm used in this study is also a CART decision tree [45]. The objective function of XGBoost is regularized, which is beneficial to control overfitting and further improving the model performance. XGBoost can effectively support parallel computing and improve efficiency. In addition to the same three parameters used with the RF model, XGBoost also adjusts other parameters, including the minimum sum of instance weight needed in a child (min_child_weight), the minimum loss reduction required to make a further partition on a leaf node of the tree (gamma), the subsample ratio of the training instances (subsample), and the parameter for column subsampling (colsample_bytree).

### 2.8. Stacking Ensemble Method

In contrast to bagging and boosting methods, stacking methods usually intend to use the heterogeneous learner as the base learner. The principle of stacking is to train different base learners and use the predicted results of the base learners as input to train the meta-learner to get the final result. In the present study, we used LR, RF, and XGBoost as base learners and a new LR model as the meta-learner to construct an ensemble model based on stacking. All the base learners obtained the best feature subset based on RFECV and they were hyperparametric optimizations and evaluations using nested cross-validation (external repeated 10 times 5-fold and internal 5-fold), as shown in Figure 2(a).

The following are the main steps of stacking (Figure 2(b)):

  Step 1. Implement a *K*-fold cross-validation to separate the training set in to *k*-folds.
  Step 2. Hold out one of the folds as validation set and train multiple independent base models to the other folds.
  Step 3. Predict the validation set using the base models.
  Step 4. Repeat the above steps to obtain the prediction results of all the base learners.
  Step 5. All the predicted results are combined into a training set as features, which is used as a new input to train the meta-learner.
  Step 6. Predict the final output using the meta-learner.

### 2.9. Model Construction

Our work consisted of four sections altogether. First, we preprocessed the cohort data. Second, we determined the algorithms to be used according to previous literature reviews and research purposes, including LR, RF, and XGBoost. We constructed these learners using default parameters and selected the best feature subsets using RFECV for each learner. Third, we trained, optimized, and evaluated three learners based on the best feature subsets for each learner. In the end, we built a proposed stacking method based on optimized base learners (Figure 3).

A pipeline was constructed to combine each component of model construction, including imbalanced data processing, model training, hyperparameter tuning, and model evaluation.

The process of the pipeline is as follows (Figure 4):

  Step 1. The data were randomly divided into five folds, of which four folds were used as the training set and one-fold was used as the test set.
  Step 2. Synthetic minority oversampling technique (SMOTE) was used to conduct imbalanced data processing for each training set.
  Step 3. Defined the hyperparametric search space and used a random-search algorithm with 5-fold cross-validation to determine the best combination of parameters for each model.
  Step 4. The best combination of parameters was applied to each algorithm and its effectiveness was evaluated on a test set.
  Step 5. The proposed stacking model was constructed by models in Step 4, and it was evaluated by a test set.

We evaluated and compared the effects of each base learner and the proposed stacking method using the same cross-validation dataset. A paired *t*-test was used to test the statistical difference of model performance.

There were two things to note here. First, we used stratified 5-fold cross-validation to divide the dataset. It was used to keep the proportion of people with and without GDM in each fold consistent with the original dataset. In addition, the data showed that the sample of women with GDM was far smaller than that of women without GDM, indicating an imbalanced dataset. Thus, we used SMOTE, an oversampling approach, to handle this problem. Different from previous studies that have realized oversampling with replacement (random oversampling) [46], the SMOTE changes the distribution of imbalanced data by creating synthetic samples among minority samples [47]. For classifying imbalanced data, the SMOTE not only improves the performance of the classifier but also alleviates the overfitting problem. SMOTE has been widely used to solve the issue of imbalanced data in the field of medicine [48, 49].

Construction and evaluation of all models were performed by the Python 3.7.0 scikit-learn library [50] and the XGBoost library (https://xgboost.readthedocs.io/en/latest/python/index.html). The stacking method was based on mlxtend 0.20.0 library (http://rasbt.github.io/mlxtend). The paired *t*-test was based on SPSS.

### 2.10. Model Evaluation

The effectiveness of the model is measured by the following metrics, including AUC, accuracy, sensitivity, specificity, and error rate. The models' accuracy, sensitivity, specificity, and error rate were calculated based on a default threshold of 0.5 and the calculation formula is as follows:

(1) $$\begin{array}{c} \text{Accuracy}=\frac{\text{TN}+\text{TP}}{\text{TN}+\text{FN}+\text{TP}+\text{FP}}, \end{array}$$

(2) $$\begin{array}{c} \text{Sensitivity}=\frac{\text{TP}}{\text{TP}+\text{FN}}, \end{array}$$

(3) $$\begin{array}{c} \text{Specificity}=\frac{\text{TN}}{\text{TN}+\text{FP}}, \end{array}$$

(4) $$\begin{array}{c} \text{Error rate}=\frac{\text{FP}+\text{FN}}{\text{TN}+\text{FN}+\text{TP}+\text{FP}}. \end{array}$$

True positive (TP) represents the number of GDM cases correctly predicted by the model. False positive (FP) represents the number of cases that the model predicts as GDM but are actually non-GDM. True negative (TN) is the number of non-GDM cases correctly predicted by the model. False negative (FN) represents the numbers of cases that the model predicts are non-GDM but are actually GDM.

## 3. Results

### 3.1. Participants' Characteristics

Table 1 shows the statistically different characteristics between participants with and without GDM. A total of 967 (14.12%) developed GDM. There were significant differences in age (*p* < 0.001) and BMI (*p* < 0.001) between the participants with GDM and those without GDM. Level of education (*p*=0.044) and personal (*p* < 0.001) and household (*p*=0.001) annual income were different between the participants with and without GDM. Behavioral factors, such as moderate physical activity, intake of unsaturated fatty acids, and dietary supplements, also differed between the two groups (*p* < 0.05). From the perspective of disease history and family history, those with GDM had different histories in terms of GDM, hypertension, uterine fibroids, hysteroscopic surgery, diabetes mellitus in first-degree relatives (FDRs), and stroke in second-degree relatives (SDRs) than those without GDM (*p* < 0.05). However, no significant differences were found in sleep quality, depression status, dietary habits, vigorous and mild physical activity, smoking before pregnancy, alcohol intake, abortion, and parity between the two groups.

### 3.2. Optimal Features Subset and Models Performances

The RFECV method based on the LR, RF, and XGBoost algorithms selected 71, 26, and 5 features, respectively. The XGBoost model required the least number of features, including age, BMI, renovation of the living environment, gravidity, and SDRs stroke history. The optimal feature subset of the three models is shown in Table 2.

Figure 5 shows the average performance of the three models after feature selection and hyperparameter adjustment. In general, the RF and XGBoost models performed slightly better than the LR model. The RF model had the highest average accuracy, specificity, and lowest average error rate among the three base models. The average accuracy and average specificity of the RF model reached 0.638 (95% confidence interval (CI) 0.628–0.648) and 0.683 (0.669–0.698), respectively. The average error rate of RF was 0.362 (0.352–0.372). The XGBoost model had the best average AUC and sensitivity. The average AUC and sensitivity of the XGBoost model reached 0.618 (95% CI 0.612–0.623) and 0.601 (0.582–0.620), respectively.

In order to optimize the effectiveness of the models, we combined the three models with an additional LR algorithm by the stacking ensemble method. The stacking ensemble method was able to consider the best hyperparameters for the three models as well as the best subset of features. Figure 5 shows that the simple stacking technique led to an improvement in the average accuracy and specificity of the models, reaching 0.666 (95% CI 0.663–0.670) and 0.725 (0.721–0.729).It had the lowest average error rate of 0.333 (0.330–0.337). To test the statistical significance of differences among classifiers, a paired samples *t*-test is performed regarding the RF and stacking method. We selected RF because it showed the best average accuracy, specificity, and lowest error rate.  Table 3 shows that the differences between the stacking method and RF were statistically significant (*p* < 0.001).

### 3.3. Feature Importance Ranking of the Three Models

Figure 6 shows the ranking of the top 10 important features of the LR model and RF model. The importance ranking of the five features included in the XGBoost model is also presented in Figure 6. The family history of hypertension in FDRs, unplanned pregnancy, and family history of stroke in SDRs were the most important features in the LR, RF, and XGBoost models, respectively. Abortion, soybean oil intake, and probiotic intake were predictive in the LR and RF models. Renovation of the living environment during the year was a significant predictor of the RF and XGBoost models. Only age had a strong predictive effect in all three models.

## 4. Discussion

We proposed a stacking ensemble method using LR, RF, and XGBoost algorithms for predicting GDM risk in women in the first trimester. We only used the easily available predictors, such as sociodemographic factors, lifestyle and behavioral factors, environmental factors, dietary habits, supplement intake, personal, and family history of disease. This method is designed to help women who live in areas with inadequate medical resources or who cannot get regular prenatal care. The pathophysiology of GDM is complex and most prior research has relied on biochemical markers factors to identify those who are at risk of developing the disease [15, 16, 31]. However, women in low and middle-income countries tend to have a severe disease burden of GDM, and the development of more concise and easy-to-use models is warranted [51].

Our results showed that the stacking model achieves the best accuracy and specificity as well as the lowest error rate. This finding is similar to the results of the previous studies, and stacking could yield better results in predicting the onset of diabetes such as GDM [52]. In the present study, we also compared the performance of our stacking method with that of the RF, and the results of the statistical test showed that the stacking method was better than the RF in these three metrics. The bagging algorithm, such as RF, is a good example of homologous ensembles. Its main components are the parallel combinations of numerous weak classifiers, which output the final result via a voting or averaging approach. In this process, the dataset needs to be resampled based on different sample distributions and each weak classifier is built from each bootstrap samples. Stacking is a classic example of heterogeneous ensembles. In this method, a variety of independent base learners with strong performances are used to predict in the first layer, and the prediction result of each base learner is used as the input of the meta-learner. The final prediction result is obtained through the meta-learner in the second layer [53]. Because of its unique way of working, stacking offers greater flexibility than bagging methods and allows for better prediction results by setting up different base learners and meta-learners to reduce variance and bias [54, 55]. It is worth noting that bagging can be incorporated into the framework of stacking as a base learner. In our study, RF and XGBoost were used as the base learners for stacking methods. The popular stacking framework has theoretically demonstrated that the ensemble results of stacking should be better or asymptotically equivalent to the optimal base learner in its first layer [56]. What was more, we constructed different base learners using their respective optimal feature subsets. Previous studies have suggested that attribute partitioning methods generally improve independence and result in better model performance than data partitioning [57, 58].

We explored the order of feature importance for three base learners. Combined with the ranking of the feature importance in the final model output, age, BMI, alcohol intake, intake of unsaturated fatty acids such as soybean oil, probiotic intake, moderate to vigorous physical activity, passive smoking, household size, family history of hypertension in FDRs, and stroke in SDRs, renovation of the living and working environment, unplanned pregnancy, abortion, and gravidity were significant predictors worth noting. For one thing, the differences of age, BMI, physical activity, intake of unsaturated fatty acids, and other factors between the GDM cases and non-GDM cases in this study were statistically significant. For another thing, most of these features have been statistically confirmed to be associated with the onset of GDM. Age, BMI, dietary factors, physical activity, and abortion were significant risk factors for GDM and have also been considered significant predictors in previous predictive modelling studies [16, 59–61]. Other features, such as alcohol consumption, family history of hypertension, and passive smoking, were associated with a higher risk of GDM in Chinese women [62, 63]. However, the role of gravidity, unplanned pregnancy, and interior renovation exposure in the risk prediction model for GDM requires further validation. We did not focus on biochemical indicators in this study, although these indicators may play an important role in building a risk prediction model for GDM. Whereas, sociodemographic factors, including disease history and family history, may reflect changes in certain underlying physiological mechanisms that suggest the risk of GDM development. Machine learning algorithms could be used to identify probable disease risk factors. As a result, the study's key features may not only provide new evidence for their inclusion in future research but also reveal potential risk factors for GDM that require additional investigation. What was more, we chose RFE combined with cross-validation when selecting the optimal feature subset. The RFE method is able to obtain the subset of features that make the model perform best under specific conditions. By combining this method with cross-validation, we are able to obtain the smallest subset of features while ensuring the effectiveness of the model. This way of selecting feature subsets helps in the construction of stacking models because stacked models require the first layer of base learning equipment to have good generalization power. Feature selection simplifies the complexity of the model and reduces the running time while ensuring strong predictive performance of the base learner [58].

Our study has a number of advantages. First, our stacking model performed well in predicting the GDM of women in the first trimester, and using sociodemographic and behavioral data to build GDM prediction models is more practical and feasible in areas with limited medical resources. Second, a pipeline was built to combine the steps of imbalanced data processing, model development, optimization, and model evaluation, with nested cross-validation employed to ensure more consistent evaluation findings. Furthermore, since the sample in this study was nationwide, the results could be more representative than other Chinese models using small-scale or single-canter data. However, the out-stacked model's performance was limited compared to similar studies [64]. Our findings were similar to those of a Tanzanian study [51]. More important features should be included when creating prediction models, especially for machine learning algorithms. This does not imply including a larger number of features, but rather features that have been identified as relevant in prior models. Although we did not focus on clinical indicators in this study, other readily available indicators were lacking. Referring to similar research, several important predictors such as sedentary time, abdomen circumference at inclusion, and irregular menstruation were omitted in our study [59, 64]. This may be one of the reasons for the slightly unfortunate performance of our model. What was more, using more complex methods may be able to further enhance the performance. In the future, we will discuss other feature selection methods and use more complex learners, such as deep neural networks, to improve the proposed stacking method. Although nested cross-validation provides some assurance of model stability, our machine learning models still require external validation in the future.

## 5. Conclusion and Future Work

Overall, it is feasible to construct a GDM prediction model for women in the first trimester based on easily available factors by using the stacking ensemble method. Our proposed stacking method based on easily available factors has better performance than the base learners, such as RF. Our proposed approach could also be considered in other health domains, such as type 2 diabetes, hypertension, and stroke. These diseases have similar risk factors and predictors of GDM and are greatly influenced by lifestyle and behaviors. Stacking provides better results than a single learning device and is more flexible than bagging and boosting and using different subsets of features can reduce the complexity of stacking models. Therefore, future research can explore more feature selection methods and build stacking models in combination with other different base learners.

## Figures and Tables

**Figure 1:** Flowchart illustrating data cleaning and processing.

**Figure 2:** Work flow for the stacking method. (a) The structure of the proposed stacking method. (b) The principle of the stacking method.

**Figure 3:** Work flow illustrating the predictive model construction process.

**Figure 4:** Pipeline for training, optimizing, and evaluating models.

**Figure 5:** Boxplot of performance for the three models with the optimal parameter and stacking method.

**Figure 6:** Feature importance ranking of three models.

**Table 1:** Characteristics between gestational diabetes mellitus (GDM) and non-GDM groups, *N* (%).

Feature		Non-GDM group (*N* = 5,881)	GDM group (*N* = 967)	*P* value
Age group (years)	<25	1,353 (23.0)	101 (10.4)	<0.001
	25–30	2,957 (50.3)	475 (49.1)	
	>30	1,571 (26.7)	391 (40.4)	

Body mass index (kg/m^2^)	<18.5	825 (14.0)	77 (8.0)	<0.001
	18.5–24.0	3,798 (64.6)	587 (60.7)	
	>24.0	1,258 (21.4)	303 (31.3)	

Educational level	Primary school and below	30 (0.5)	6 (0.6)	0.044
	Junior and senior high school	2,084 (35.4)	299 (30.9)	
	University	3,408 (57.9)	593 (61.3)	
	Masters' degree and above	359 (6.1)	69 (7.1)	

Education level of partner	Primary school and below	29 (0.5)	10 (1.0)	<0.001
	Junior and senior high school	2,226 (37.9)	292 (30.2)	
	University	3,275 (55.7)	589 (60.9)	
	Masters' degree and above	351 (6.0)	76 (7.9)	

Occupation	No^†^	1,662 (28.3)	224 (23.2)	0.001
	Yes	4,219 (71.7)	743 (76.8)	

Occupation of partner	No	463 (7.9)	54 (5.6)	0.015
	Yes	5,418 (92.1)	913 (94.4)	

Personal annual income (10000 CNY)	<5	3,655 (62.1)	517 (53.5)	<0.001
	5–10	1,754 (29.8)	347 (35.9)	
	>10	472 (8.0)	103 (10.7)	

Household annual income (10000 CNY)	<10	3,199 (54.4)	463 (47.9)	0.001
	10–20	1,810 (30.8)	335 (34.6)	
	>20	872 (14.8)	169 (17.5)	

Household size	1–3	3,230 (54.9)	588 (60.8)	0.003
	4	1,332 (22.6)	188 (19.4)	
	≥5	1,319 (22.4)	191 (19.8)	

Moderate physical activity	No	5,074 (86.3)	858 (88.7)	0.043
	Yes	807 (13.7)	109 (11.3)	

Vitamin without vitamin D	No	3,277 (55.7)	505 (52.2)	0.046
	Yes	2,604 (44.3)	462 (47.8)	

Vitamin D	No	4,480 (76.2)	683 (70.6)	<0.001
	Yes	1,401 (23.8)	284 (29.4)	

Calcium	No	4,162 (70.8)	644 (66.6)	0.010
	Yes	1,719 (29.2)	323 (33.4)	

Soybean oil intake	No	4,029 (68.5)	711 (73.5)	0.002
	Yes	1,852 (31.5)	256 (26.5)	

Olive oil intake	No	5,338 (90.8)	853 (88.2)	0.015
	Yes	543 (9.2)	114 (11.8)	

GDM history	No	5,872 (99.8)	959 (99.2)	0.001
	Yes	9 (0.2)	8 (0.8)	

Unplanned pregnancy^‡^	No	4,203 (71.5)	734 (75.9)	0.005
	Yes	1,678 (28.5)	233 (24.1)	

Hypertension history	No	5,841 (99.3)	951 (98.3)	0.003
	Yes	40 (0.7)	16 (1.7)	

Uterine fibroids	No	5,796 (98.6)	935 (96.7)	<0.001
	Yes	85 (1.4)	32 (3.3)	

Hysteroscopic surgery	No	5,841 (99.3)	954 (98.7)	0.047
	Yes	40 (0.7)	13 (1.3)	

FDRs (diabetes)	No	5,689 (96.7)	905 (93.6)	<0.001
	Yes	192 (3.3)	62 (6.4)	

SDRs (stroke)	No	5,838 (99.3)	967 (100.0)	0.014
	Yes	43 (0.7)	—	

^†^No, no full-time job; ^‡^Unplanned pregnancy, was this pregnancy an unplanned pregnancy?

**Table 2:** Optimal feature subsets with three models.

Model	Features' list
LR	(i) Sociodemographic factors: age, ethnic minority, occupation of partner, and personal annual income.
	(ii) Lifestyle and behavioral factors: moderate physical activity, ventilator physical activity, smoking before pregnancy, smoked within the last month, drinking, cooking, and BMI.
	(iii) Environmental factors: living environmental pollution (including sewer, dumpster, and chemical, pesticide) and work environmental pollution (including noise, high temperature, heavy metal, and hair dye).
	(iv) Dietary habit and supplement intake: unsaturated fatty acids (including soybean oil, olive oil, and linseed oil); vitamins (including vitamin D and other types of vitamins); calcium, iron dietary supplement, and probiotics.
	(v) Previous pregnancy status: parity, GDM, hypertensive disorders complicating pregnancy, preeclampsia, placental abruption, late abortion, small for gestational age, premature delivery, and stillborn fetus.
	(vi) Personal disease history: hypertension, hyperlipidemia, hyperthyroidism, anemia, heart disease, chronic glomerulonephritis, cancer, epilepsy, tuberculosis, viral hepatitis type B, infertility, cervical intraepithelial neoplasia, uterine fibroids, ovarian cyst, gonorrhea, systemic lupus erythematosus, ulcerative colitis, and Sjogren syndrome.
	(vii) Family disease history: FDRs disease history (including hypertension, diabetes, hyperlipidemia, and cancer) and SDRs disease history (including diabetes, hyperlipidemia, stroke, and cancer).
	(viii) Gynecological surgery history: myomectomy, oophorocystectomy, hysteroscopic treatment, extrauterine pregnancy, diagnostic-curettage, and abortion.

RF	(i) Sociodemographic factors: age, education level, education level of partner, personal annual income, household annual income, and household size.
	(ii) Lifestyle and behavioral factors: mild physical activity, sleep quality, depression level, and BMI.
	(iii) Environmental factors: passive smoking, noise pollution of living environment, renovation (working and living environment), and cooking.
	(iv) Dietary habit and supplement intake: unsaturated fatty acids (including soybean oil, peanut oil, and sunflower oil), dietary habit, vitamins (excluding vitamin D), calcium, and probiotics.
	(v) Previous pregnancy status: parity, unplanned pregnancy, and gravidity.
	(vi) Gynecological surgery history: abortion.

XGBoost	(i) Sociodemographic factors: age
	(ii) Lifestyle and behavioral factors: BMI
	(iii) Environmental factors: renovation (living environment)
	(iv) Family disease history: SDRs having stroke
	(v) Gynecological surgery history: gravidity

**Table 3:** The paired samples *t*-test between the stacking method and RF.

	Mean	Standard deviation	Standard error mean	95% confidence interval of the difference		*t*	d*f*	*P* value
				Lower	Upper			
Accuracy (stacking-RF)	0.028	0.035	0.005	0.018	0.038	5.709	49	<0.001
Specificity (stacking-RF)	0.041	0.049	0.007	0.027	0.056	5.951	49	<0.001
Error rate (stacking-RF)	−0.028	0.035	0.005	−0.038	−0.018	−5.709	49	<0.001

A value of *p* < 0.05 was considered significant.

## Data Availability

The data used to support the findings of this study are available from the corresponding author upon request.
